# Defending against Internal Attacks in Healthcare-Based WSNs

This article has been retracted.

**DOI:** 10.1155/2021/2081246

**Published:** 2021-12-15

**Authors:** Zhe Wei, Shuyan Yu, Wancheng Ma

**Affiliations:** ^1^School of Computer Science, Civil Aviation Flight University of China, Guanghan 618307, China; ^2^Shaoxing University Yuanpei College, Shaoxing 312000, China

## Abstract

In view of the spatiotemporal limitations of traditional healthcare services, the use of wireless communication has become one of the main development directions for the medical system. Compared with the traditional methods, applying the potential and benefits of the wireless sensor networks has more advantages such as low cost, simplicity, and flexible data acquisition. However, due to the limited resources of the individual wireless sensor nodes, traditional security solutions for defending against internal attacks cannot be directly used in healthcare based wireless sensor networks. To address this issue, a negative binomial distribution trust with energy consideration is proposed in this study. The proposed method is lightweight and suitable to be operated on the individual healthcare sensors. Simulations show that it can effectively deal with the internal attacks while taking the energy saving into consideration.

## 1. Introduction

In the healthcare and medical field, due to the small size of individual sensor nodes in the wireless sensor networks (WSNs) and the adoption of wireless communication technology, compared with fixed healthcare equipment, these sensor nodes have the advantages of portability, real-time monitoring, and ease of positioning, so they can be used for remote health monitoring, first aid, etiological diagnosis, drug management, and other healthcare needs [1, 2]. Even with the help of these WSN nodes, patients are free of home activities and will not affect the healthcare treatment, as long as they are within the sensing range of WSNs. In addition, it is convenient for the nursing staff to understand the patient's vital signs data in real time such as blood pressure, blood oxygen, body temperature, heart rate, ECG, and respiration, so as to further analyze the patient's healthcare condition and give feedback in time. WSNs are now becoming one of the most promising technologies to achieve the e-health, which is defined as the application of Internet and other related technologies such as IoTs in the healthcare industry to improve the access, efficiency, effectiveness, and quality of clinical and business processes utilized by healthcare organizations, practitioners, patients, and consumers to improve the health status of patients [3–6].

However, due to the limitations of energy consumption, storage, and processing capacity of the individual wireless sensor nodes, some security technologies currently used in wired networks or traditional wireless networks cannot be directly applied to healthcare based WSNs. Therefore, it is necessary to develop new security technologies or modify existing security mechanisms to make them suitable for such networks. Two main challenges in the security design of healthcare based WSNs are as follows. (1) Sensor node itself is limited in computing power, storage space, communication bandwidth, and power supply, and usually large amounts of healthcare related data needs exchanging between these sensor nodes. Therefore, if complex encryption algorithms and protocols are used in the security solutions, even if they can be implemented on the individual nodes, their operation will accelerate the energy consumption of nodes and shorten their normal services. (2) Since the communication channel of wireless sensor network is open, any internal devices can easily monitor the information exchanged by nodes in the network as long as the communication interface is configured with the same frequency. In addition, it is not complicated to destroy the availability of wireless channel or conduct electronic interference to the channel from the technical point of view. Thus security and energy consumption are two important issues for WSN deployment in the healthcare applications.

The main contribution of this study is as follows. To address the above security and energy issues for the healthcare based WSNs, a negative binomial distribution trust with energy consideration is proposed in this study. Compared with traditional trust methods, the proposed method is lightweight and suitable to be operated on the individual healthcare sensors, and it can effectively deal with the internal attacks such as the selective forwarding attack. Besides, unlike traditional methods, the proposed method takes the energy as part of the trust so that the energy of the individual nodes can be balanced and the service provided by the network is accordingly prolonged.

The rest of this paper is organized as follows. Firstly, this research studies and analyzes the current status quo of WSNs security issues, discusses and analyzes the internal causes of network attacks, and studies and summarizes the main types of attacks on the network and related preventive measures. Secondly, this paper gives an overview of reputation and the trust mechanism in WSNs, which is an important supplementary tool for the network security. It discusses the background, significance, concept and characteristics of reputation and trust, the composition of reputation, and trust system. Thirdly, the negative binomial trust method that was proposed in our previous work is introduced and its advantages over the traditional trust methods are discussed. Then, based on the negative binomial trust and energy consideration, to defend against the internal attacks in healthcare based WSNs, our proposed method is presented and related simulation tests are also showcased. Lastly, conclusions are drawn and future study is pointed out.

## 2. Background

### 2.1. Security Issues

The security problem of wireless sensor networks has been widely concerned by scholars. The authors in [7] comprehensively discuss the impact of DoS attacks on wireless sensor networks as well as the countermeasures and point out that these attacks are all originated from the security vulnerabilities of individual sensor nodes in their physical layer, data link layer, network, and transport layer. The authors also summarize the necessity of adding security protection mechanism in wireless sensor network routing design stage. In [8], an enhanced dynamic resource routing protocol is proposed. In this protocol, individual nodes that act in a hybrid monitoring manner use the passive ACK mode to observe the communication between other nodes in the network. These nodes then classify the nodes participating in the communication according to the observed communication results, which helps to build a trusted routing path from the source to the destination. In order to prevent nodes from receiving false public keys from malicious nodes, a trust based secure public key authentication service model is proposed in [9]. The nodes in the network not only use their private keys to digitally sign the public keys of other nodes to build a trusted network but also monitor other nodes, build trust tables, and store them locally. Most of the above researches focus on external security attacks of wireless sensor networks. However, there is little discussion on internal attacks from internal nodes, such as malicious nodes' attacks and damage to the network. In addition, because the malicious nodes can still access the network and hold the relevant secret key information, it is unable to effectively protect the network from attacks from the inside of the network only by relying on security technology.

The authors in [10] study and discuss how to add security mechanisms to cluster based communication protocols in wireless sensor networks and propose an improved LEACH protocol, i.e., SLEACH. On the premise of preserving the core part of LEACH algorithm, the main framework of SPIN that is based on the symmetric secret key method is added to LEACH protocol to ensure the security and reliability in the dynamic formation process of clusters.

Most reputation or trust systems assume that the node ID remains unchanged throughout its work cycle and predict the future behavior results based on the results of the past historical behavior of the node. In practical application, with the decreasing reputation of some nodes, it is very likely to change their ID, which can wash away their past malicious behaviors. The authors in [9] have made a more in-depth analysis and discussion on the impact of this ID conversion problem in the reputation system and propose a trust mechanism based on partial identity information, that is, the trust system based on partial characteristic information of nodes.

In order to ensure the effectiveness and security of specific data transmitted by wireless multimedia sensor networks, especially in data fusion, to prevent the system from being destroyed by the damaged data fusion nodes, a security method based on digital watermarking was proposed in [11]. The authors in [11] embed the secret data generated by the antiattack watermarking algorithm into the image data, and the secret data is transparent to the data fusion node. The data fusion node can fuse the original image data without detecting the existence of the secret data, and only the base station node can extract the encrypted number from the final data received by the base station node. The authors in [12] proposed an end-to-end data authentication method in wireless sensor networks based on digital watermarking method. In this method, the authentication data is superimposed with the sensing data of the node as a digital watermark. When the final data reaches the base station, the base station verifies the effectiveness of the watermark information to authenticate the final data. It can be seen that, in this method, the watermark information is only added in the data source and finally verified by the base station.

From the perspective of data fusion in wireless sensor networks, the authors in [13] study and describe the security problems and corresponding measures in the single hop and point-to-point data fusion especially in the initial phase, data fusion phase, data authentication phase, and data recovery phase. Since the encryption and the authentication operations involve the secret key, the establishment of the secret key is the first step to establish the security infrastructure. From the perspective of secret key management, the authors in [14] discuss the establishment mechanism of secret key in wireless sensor networks in detail and also make some research and analysis on the intrusion detection and the coping strategies that destroy the network functions.

### 2.2. Attacks and Preventive Measures

Several common attacks in healthcare based wireless sensor networks are listed in this section, and the corresponding preventive measures are studied and discussed.

#### 2.2.1. Sybil Attack

In Sybil attack, a single node has multiple illegal false identities in the network. Sybil attack first appeared in the research of P2P network and then appeared in ad hoc wireless sensor network [15]. Some networks adopt fault-tolerant mechanisms such as distributed storage. These methods assume that the nodes in the network are distributed and different. In fact, a single malicious node can impersonate multiple nodes; that is, it has multiple identities. Therefore, Sybil attack will greatly reduce the performance of these fault-tolerant mechanisms. In addition, Sybil attack will also greatly damage routing protocols based on geographical location, because these routing protocols will involve the use of location coordinates of multiple different nodes [16].

The common preventive measure of Sybil attack is the channel detection method [17]. In this method, each node assigns its neighbor node a unique communication channel, which is to detect whether the neighbor node can communicate with the node through a given channel. Because a sensor node cannot receive or send data in two or more channels at the same time, if the corresponding neighbor node's communication is not received on a given channel, it often means that Sybil attack may occur [14].

#### 2.2.2. Sinkhole Attack

In the sinkhole attack, an attacker tries to attract all the traffic in a certain subarea, which makes the attacker have the opportunity to tamper with and destroy some interesting data in this traffic [18]. Sinkhole attack usually takes the way of attacking a node in the network first and then uses deception to claim that the node can provide high-quality routing to the base station node, which makes the node attractive to the surrounding nodes in routing. Due to its special communication mode, wireless sensor networks are very vulnerable to sinkhole attacks, because the data packets transmitted by all nodes generally have the same destination address, that is, the address of the base station. Once a malicious node claims to provide a high-quality routing way to other nodes, it can attract a large number of network nodes [16]. Another way of sinkhole attack is to select forwarding data packets; that is, malicious nodes can selectively forward these packets after attracting the surrounding data traffic.

Generally, the route to the base station through the sinkhole attack area is more attractive and more frequently used, which means that the nodes in the sinkhole attack area lose energy quickly and form an energy hole. According to this principle, [18] proposed two solutions to sinkhole: (a) The base station samples the residual energy of nodes in each sensing area by using geographical statistics method and judges the possibility of sinkhole attack according to the statistical evaluation data after sampling. If it is determined as a sinkhole attack, the base station informs all nodes to avoid this area when routing. (b) A distributed detection method is used to detect which areas have low residual average energy to determine whether a sinkhole attack has occurred.

#### 2.2.3. Wormhole Attack

In the wormhole attack, an attacker secretly sets up a low latency data channel at two distant points and replays the data at another point [19]. By launching a wormhole attack, the attacker can also claim that it is very close to a node with only a few hops away, while the actual distance can be very far. In addition, the wormhole attack will disturb the network topology structure, which makes the nodes that are far away from each other in geographical location mistakenly as neighbor nodes. The wormhole attack also makes it difficult for network nodes to find routing paths with only a few hops, which in fact has a great harm to the network routing protocol.

A more effective preventive measure against the wormhole attack is to use the location-based secret key distribution mechanism [20]. In this mechanism, the data packets sent by sensor network nodes are authenticated by the location-based secret key, so as to avoid passing the data packets to the next hop node far away from the location.

#### 2.2.4. Select Forwarding Attack

In wireless sensor networks, malicious nodes will refuse to forward received data packets and discard these packets. In addition, in order to avoid the neighbor nodes aware of their malicious behavior and bypass the malicious node, such malicious nodes will have a choice of forwarding partial packets and discard the remaining packets [21]. By using selective forwarding attack, the attacker can successfully interrupt the normal operation of the network, especially when the attacker is close to the base station, and the harm of this kind of attack will be more serious. Compared with other attacks, selective forwarding attacks are more difficult to detect because normal nodes in the network will occasionally drop data packets due to network congestion [16].

For selective forwarding attack, one more effective preventive measure is to use neighbor node supervision mechanism. In [22], the network node uses hybrid monitoring mode to supervise its neighbor nodes, and it is stipulated in advance that the number of data packets received by a node in the network should be equal to the number of packets forwarded by the node. When the number of data packets received and transmitted by a node in the network is different, the node may be a malicious node, and the other members of the network will eventually jointly judge the suspected node.

## 3. Reputation and Trust Mechanism

Reputation and trust mechanism is a kind of soft security method [23, 24]. Soft security usually refers to the use of social or group methods to restrict and control individual behavior, while hard security mainly refers to traditional security methods such as authentication mechanism and authorization mechanism. Generally, the main difference between the two security mechanisms is how to deal with illegal intrusion in a system. The purpose of hard security is to prevent intruders from entering the system; that is, there should be no illegal intruders in the system [25–27]. Soft security, such as reputation and trust mechanism, allows the existence of intruders in the system to a certain extent, but this method attempts to identify the intruders and prevent them from destroying the system or to minimize the degree of damage [28–31].

In wireless sensor networks, nodes can increase or lose their trust value according to the completion of specified tasks and the behavior of nodes. In addition, only when the trust value of the node is higher than the predefined threshold value can it participate in the task request initiated by other nodes in the network. Therefore, the reputation and trust mechanism can be used to evaluate the ability of nodes to complete the specified tasks, and trust information can be used to make decisions [32–34].

There is no unified definition of reputation and trust. It is generally believed that trust is essentially a kind of belief, which is the degree of credibility of other entities' future behavior held by an entity based on its own past experience. Therefore, from this perspective, trust has a certain degree of subjectivity [35–39]. Reputation is the trustor's trust in the trustee. In [39], reputation consists of direct experience and witness information. When a trustee asks a neighbor node about the trustor's reputation information, if the neighbor node has ever made a transaction with the trustee, the neighbor node will feedback the trustor's reputation information about the trustee, which is called testimony as direct experience. When the neighbor node has not dealt with the trustee, the neighbor node will return a list of its own neighbors to the trustee, which is called reference table as witness information. In addition, the reputation of an entity is based on the trust held by other nodes, which is a global perception about the behavior of the node. From this perspective, reputation has certain objectivity. Similar to [40], this study does not make a strict distinction between reputation and trust in terms of concept, and the two concepts have not obtained consistent distinction in academic field.

Generally, a trust system consists of five parts [40]: information collection, information evaluation, entity selection, transaction execution, and reward and punishment mechanism. Information collection is responsible for collecting historical behavior information of entities in the reputation system. The source of historical behavior information can be direct experience or indirect experience or recommended information provided by other entities. When the historical reputation information of an entity is collected, it can be regarded as input information and input into the reputation calculation engine (model) for calculation, and the calculation results are used as the reputation evaluation of the corresponding entity. According to the results of the previous evaluation system, the appropriate entity is selected to trade with, and, in the actual process, node with the highest trust is selected. In addition, the transaction execution in wireless sensor networks can be the transmission of data packets between nodes, routing information response and request, data query, and so on. After the transaction is completed, the customer entity shall reward or punish the service entity according to the service quality provided by the service entity or the transaction result after the completion of the transaction. According to [40], the components of a trust system are presented in Figure 1.

## 4. Negative Binomial Trust

The trust mechanism depends on the historical records of participating nodes, and Bayesian theory that attempts to discover the behavior patterns through historical actions fundamentally complies with the procedure of the trust evaluation. Instead of using binomial distribution based trust [41], negative binomial distribution based trust has many distinctive features such as energy efficiency. In our previous work [42], we proposed a negative binomial distribution based trust that can well be applied in WSNs. A simple deduction of it, on which our proposed method is mainly based, is presented as follows.

Consider a sequence of independent Bernoulli trials with success probability *ρ*, and let *Z* denote the number of failures until the rth success. Random *Z* is called the negative binomial random variable with parameters *ρ* and *s*. Its probability mass function is defined by

(1) $$\begin{array}{c} P\left(Z=s|r,\rho \right)==\left(\begin{array}{c} r+s-1\\ s \end{array}\right)\rho^{r}{\left(1-\rho \right)}^{s}, \end{array}$$

where *s* = 0,1,2... and 0 < *ρ* < 1.

This is the probability of observing *s* failures before the *r*th success or *s* + *r* trails are needed until the *r*th success to take place. In (1), *ρ* is the binomial success probability and its conjugate prior distribution is beta distribution. Next, consider the posterior of *ρ*.

(2) $$\begin{array}{c} P\left(\rho |Z\right)=\frac{P\left(Z|\rho \right)P\left(\rho \right)}{\int P\left(Z|\rho \right)P\left(\rho \right)d\rho }\\ =\frac{\Gamma \left(\alpha +\beta +r+s\right)}{\Gamma \left(\alpha +r\right)\Gamma \left(\beta +s\right)}\rho^{\alpha +r-1}{\left(1-\rho \right)}^{\beta +s-1}. \end{array}$$

It indicates that posterior *P*(*ρ* |*Z*) has a beta distribution with parameters *a* + *r* and *β* + *s*. Thus, the expectation of *ρ* is defined by

(3) $$\begin{array}{c} E\left(\rho \right)=\frac{\left(\alpha +r\right)}{\left(\alpha +\beta +r+s\right)}. \end{array}$$

In (3), *E*(*ρ*) can usually be regarded as the trust value of the participating nodes in some activities such as routing information response, while *α* and  *β*  can be regarded as the amounts of cooperation (positive evaluation) and noncooperation (negative evaluation) in these activities, respectively. *α* and  *β*  are also called shape parameters, and a shape parameter is any parameter of a probability distribution that is neither a location parameter nor a scale parameter. Further, there are three possible cases for the outcome of (3); namely,

(4) $$\begin{array}{c} E\left(p\right)=0.5,if\left(\alpha +\;r\right)=\left(\beta +s\right). \end{array}$$

When the shape parameters *α* and  *β* in the beta distribution are equal, this indicates that the amounts of cooperation and noncooperation of a node in an activity or transaction are the same, and the trust value of the node is 0.5. In most literatures, the threshold of the trust value is 0.5. It is generally believed that the node with trust value of 0.5 is a neutral node which does not belong to illegal node or malicious node.

(5) $$\begin{array}{c} E\left(p\right)>0.5,\left(\alpha +\;r\right)>\left(\beta +s\right). \end{array}$$

When the shape parameter *α* in the beta distribution is greater than *β*, it indicates that the amount of cooperation is greater than that of noncooperation in an activity or transaction. At this time, the trust value of the node is greater than 0.5. It is believed that the larger the value is, the higher the trust and credibility of the node will be.

(6) $$\begin{array}{c} E\left(p\right)<0.5,if\left(\alpha +\;r\right)<\left(\beta +s\right). \end{array}$$

In this case, the trust of the node is less than 0.5. Generally, the node will be marked as malicious or illegal. In the trust system, once a node is identified as being malicious, other nodes will no longer cooperate with the node, and the data received from the node will also be discarded by other nodes, which is formally equivalent to the fact that the node is isolated from the network.

In the traditional binomial trust, to monitor and save the trust parameters of the observed node, the observer node should update and calculate the trust of the observed node immediately after each transaction. From the perspective of energy consumption, this frequent trust update is not conducive to the wireless sensor network nodes with limited resources. By contrast, in the negative binomial trust, the trust parameters can be computed according to the different task requirements. For example, in tasks with low time urgency, the amounts of cooperation and noncooperation of nodes can be observed and recorded within the time equivalent to *r* + *s* transactions, and then the trust is updated and calculated according to the actually observed *r* and *s*. It can be seen that, in the negative binomial trust, it is unnecessary for the observer nodes to do the trust update after each transaction, which can reduce the number of trust update calculations, so as to save the energy consumption of network nodes accordingly.

## 5. The Proposed Method

The proposed method takes the binomial trust for the trust computing, and, for energy considerations, an energy trust is integrated into the trust computing so as to balance the energy consumption.

Assume that node *j* makes a series of requests within a fixed period of time ∆*T* from node *i*. If *j* receives *r*(∆*T*) positive outcomes and *s*(∆*T*) negative outcomes from *i* within ∆*T*, then, according to the negative binomial trust, the trust value of *i* maintained by *j* is defined by

(7) $$\begin{array}{c} T_{i,j}=\frac{\alpha_{i,j}+r_{i,j}\left(\Delta t\right)}{\alpha_{i,j}+\beta_{i,j}+r_{i,j}\left(\Delta t\right)+s_{i,j}\left(\Delta t\right)}. \end{array}$$

In the application of healthcare based WSNs, ∆*T* is adjustable according to the specific scenarios. For example, during the heart rate monitoring, ∆*T* can be set as 1 so as to keep the trust updated, while in the body temperature monitoring, ∆*T* could be set larger and the trust computing needs not necessarily to be done frequently so the energy of the sensor nodes can be saved.

Further, according to [43], when transmitting *k*-bit data packet within distance *d* in wireless sensor networks, the transmitter energy consumption *E*_T_(k, d) is defined by

(8) $$\begin{array}{c} E_{T}\left(k,d\right)=\left\{\begin{array}{cc} kE_{\text{elec}}+k\varepsilon_{FS}d^{2}, & d<d_{0},\\ kE_{\text{elec}}+k\varepsilon_{MP}d^{4}, & d\geq d_{0}, \end{array}\right) \end{array}$$

where *E*_elec_ is the electronics energy such as signal coding and spreading; *ε*_FS_d^2^ and *ε*_MP_d^4^ are the amplifier energy in the free space fading channel (*d*^2^ power loss) and multipath fading channel (*d*^4^ power loss), respectively. If distance *d* is less than the predefined threshold *d*_0_, power loss can be modeled as the free space model; else, if *d* is greater than or equal to *d*_0_, power loss is modeled as the multipath model; and when receiving this *k*-bit data packet, the receiver energy consumption *E*_R_(k) is defined by

(9) $$\begin{array}{c} E_{R}\left(k\right)=kE_{\text{elec}}. \end{array}$$

Under ideal situations, high trust node should be selected for task execution such as packet relay, but, in reality, the frequent use of the same node would result in faster battery drainage and later these nodes are usually discarded. To balance the energy consumption, the residual energy is considered as part of the trust, and the energy trust is defined by

(10) $$\begin{array}{c} T_{\text{energy}}=\frac{E_{I}-E_{R}-E_{T}}{E_{I}}, \end{array}$$

where *E*_*I*_ is the initial energy; and, with the energy trust, the compound trust *T*_com_ is defined by

(11) $$\begin{array}{c} T_{\text{com}}=\omega_{1}T_{i,j}+\omega_{2}T_{\text{energy}}, \end{array}$$

where *ω*_1_ and *ω*_2_ are weights and 0 <*ω*_1_ + *ω*_2_ < 1.

## 6. Simulations

In this section, BDTMS [41] is selected as the baseline for comparison with our proposed method, namely, negative binomial trust with energy consideration (NBTEC). In BDTMS, a binomial distribution based trust scheme is proposed for healthcare-oriented WSNs. BDTMS is applicable to defend on-off attacks and bad mouthing attack; however, it does not take the energy of individual sensor node into consideration, which is not very suitable for the healthcare based WSNs especially when a large amount of data is transmitted among sensor nodes.

Suppose that 50 sensor nodes are transmitting and relaying patient body temperature readings. The temperature readings from normal sensor nodes are within 35°C∼42°C. There are 15 evenly deployed malicious nodes and 5 evenly deployed selfish nodes. For malicious nodes, they launch on-off attacks; that is, they randomly either relay data readings that they directly receive or inject false readings other than 35°C∼42°C and then transmit those modified readings to the next node. For selfish nodes, they launch selective attacks; namely, they selectively drop some or all the received data readings. In each simulation, the base station launches 250 queries to collect temperature readings from every sensor node over a fixed period of time. Each node has a unique ID, every node has the prior knowledge about the location of the base station, and sensor nodes are capable of bidirectional communication on every link. Once a node's trust is lower than 0.45, it will no longer be selected for data transmission. Further, assume that the initial trust of each node is 0.6, *E*_*I*_ = 0.5 J, *E*_elec_ = 50 nJ/bit, *d* = 1 m, and *ε*_FS_d^2^ = 10 pJ/bit/m^2^, the channel bandwidth is set to 1 Mb/s, *ω*_1_ = *ω*_2_ = 0.5, and △*T* equals a certain number of queries for the bases station, and it varies in different tests.

In this part, the data reading correctness (DRC) and the average residual energy of sensor nodes (ARE) are tested between the two methods BDTMS and NBTEC. Test results are shown in Figures 2 and 3, respectively.

In Figure 2, the DRC is the ratio of the total received correct data readings to the total received false data readings. It is obvious that the larger the ratio is, the better the network can deal with the internal attack, and a higher ARE also means that the network has the power to do more work.

To a selfish node, conserving its own internal resources like residual energy is more important than being trust qualified to take part in a certain task, while to a malicious node, it has to be trust qualified and be selected for participating a certain task, so that it has opportunities to launch attacks like injecting erroneous data readings to be relayed. Generally, once requested, each sensor node should correctly transmit its received data readings to the next node; thus both methods should have the same or similar DRCs, but when malicious nodes and selfish nodes exist in the network as shown in Figure 2, the DRC of NBTEC is always higher than that of the BDTMS; for example, at the 200^th^ query, NBTEC (△*T* = 10) has a DRC about 10, NBTEC (△*T* = 20) has a DRC about 21, and BDTMS is only around 7. This is because, in NBTEC, △*T* = 10 denotes that the trust update is done after very 10 queries, so, within these queries, more malicious behaviors can be recorded, which results in a faster malicious node detection and isolation. Then this is also the reason why when △*T* = 20, a larger DRC can be obtained in the proposed method. It can be noticed that, theoretically, the larger △*T* is, the faster the detection becomes, but the individual sensor node may not have enough memory to hold other node's behavior records within larger △*T*.

Further, the average residual energy of the two methods is tested in Figure 3. As the query number increases, the AREs of both methods drop gradually, but, compared with BDTMS, NBTEC always drops more slowly. For example, at the 200^th^ query, NBTEC has an ARE about 0.25 J, while BDTMS is around 0.21 J. The difference can be found in the trust computing of both methods. As mentioned previously, the trust update in BDTMS is done after each query, while it can be computed within certain queries in NBTEC, which helps to save the computing energy. It is also theoretically possible that the large △*T* is, the more energy can be saved, but, again, this process is subjected to the sensor's limited memory.

The number of trust qualified nodes (NTQN) is tested in Figure 4. With the increasing number of queries, the NTQN in both methods drops accordingly; at the 250^th^ query, BDTMS has an NTQN about 38, while NBTEC (△*T* = 10) is about 33 and NBTEC (△*T* = 20) is about 31. BDTMS always has a larger NTQN than NBTEC in this test. It seems to indicate that more trust qualified nodes exist in BDTMS, which is good for the network operation. It is true when there are only normal nodes in the network, but when there exist malicious nodes and selfish nodes, it deserves further analysis. Note that, in the simulation settings, there are 30 normal nodes and 20 malicious and selfish nodes. NBTEC (△*T* = 20) has an NTQN about 31 in Figure 4 and has a high DRC about 43 in Figure 2 both at the 250^th^ query which helps to explain that NBTEC can better detect the malicious nodes, resulting in more normal trust qualified nodes left. BDTMS has an NTQN about 39 at the end of query, but it has a low DRC about 8, which indicates that there still exist more malicious and selfish nodes to be detected in the network.

## 7. Conclusions

To deal with the internal attacks for healthcare based WSNs, a negative binomial distribution trust with energy consideration is proposed in this study. Compared with the binomial distribution based trust, the proposed method has high data reading correctness and a high average residual energy and can better detect the malicious nodes and defend against the internal selective forwarding attacks. When dealing with the internal attacks, trust mechanism has received much attention by researchers, but still its related study is in the initial stage. Some future research directions regarding this paper are as follows. (1) How to define the size of △*T* should be studied. Larger △*T* will inevitably affect the storage of sensor nodes, but smaller △*T* will also affect the detection effect of malicious nodes. (2) The NTQN in the proposed method cannot reach 30, meaning that some malicious or selfish nodes still exist, which is still worthy of further study.

## Figures and Tables

**Figure 1:** Five parts of a trust system.

**Figure 2:** Data reading correctness (DRC).

**Figure 3:** Average residual energy (ARE).

**Figure 4:** Number of trust qualified nodes (NTQN).

## Data Availability

The data sets in the simulation tests are assumed to be the body temperature readings, and the data readings are generated within each value interval; therefore, interested researchers can generate their own data within the two value intervals as presented in our simulation tests.
